RETRACTED

# Clinical Application of Quantitative CT Technique in Assessing Liver Fat Content in Patients with Schizophrenia

**DOI:** 10.1155/2022/7006133

**Published:** 2022-08-16

**Authors:** Mengyang Han, Yilian Lin, Hong Chen, Fang Hua, Jianye Zhang, Jinhong Wang

**Affiliations:** ^1^Department of Radiology, Shanghai Mental Health Center, Shanghai Jiao Tong University School of Mdeicine, Shanghai 200030, China; ^2^Department of Radiology, The Seventh People's Hospital of Shanghai University of Traditional Chinese Medicine, Shanghai 200137, China

## Abstract

This paper investigates the clinical application value of quantitative CT (QCT) technique in evaluating liver fat content in patients with schizophrenia. 457 patients with schizophrenia underwent abdominal CT and QCT scans. QCT postprocessing software (QCT Pro version 6.1) measures the percentage of liver fat content in all patients and calculates the average value. Then, the CT workstation displays the corresponding liver/spleen CT value ratio. SPSS 25.0 software is used for statistical analysis of data, and the correlation coefficient between the mean liver fat content. The ratio of liver/spleen CT values is calculated and the consistency between the results is compared. The ROC curve is used to define the cutoff value of the target and evaluate its diagnostic efficiency. There is a high negative correlation between the mean liver fat content and the ratio of liver/spleen CT value in all schizophrenia patients (*r* = −0.935, *P* < 0.05). The identification rate of patients with mild fatty liver by QCT technology is 4 times higher than that of the liver and spleen CT value ratio (50.98% Vs 12.47%). Taking the ratio of the liver to the spleen as the standard, the ROC curve of the liver fat content in QCT is drawn, the cutoff values of the mean liver fat content of the normal liver and mild fatty liver and mild and moderate fatty liver were 9.35% and 19.4%, respectively. Comparing this result with the results obtained by the existing QCT for the fatty liver diagnosis and grading standard value (American standard) shows that there is a difference of about 5% between the two. Compared with the semiquantitative liver/spleen ratio, QCT technology can quantify the liver fat content. Given the particularity of patients with schizophrenia, QCT can be used as an important test for identifying early fatty liver and assessing the severity of fatty liver.

## 1. Introduction

With the improvement of people's living standards and the change of dietary habits, the incidence of fatty liver is getting higher and higher [1, 2], and it has become the primary liver disease endangering the health of Chinese people. Due to unreasonable lifestyle (including substance abuse, smoking, and static lifestyle), the influence of the disease itself and antipsychotic drugs, the prevalence of fatty liver in patients with schizophrenia is higher than that of ordinary people. It occurs with the metabolic syndrome [3], so accurate measurement, diagnosis, evaluation of treatment effect, and follow-up monitoring of fatty liver are crucial. In clinical application, the common evaluation methods of fatty liver include ultrasound, magnetic resonance imaging (MRI), liver biopsy, and CT liver-spleen ratio method. In view of the particularity of patients with schizophrenia and the advantages and disadvantages of each detection method, CT examination is the main method in our hospital.

RETRACTED

In recent years, with the development of quantitative CT (QCT) technology, QCT has made great progress in evaluating fatty liver. It is particularly important to evaluate mental illnesses, especially severe mental illnesses (such as schizophrenia) that cause heavy socioeconomic and safety burdens or fatty liver caused by drugs. Therefore, this study intends to explore the correlation between the average percentage of liver fat content in patients with schizophrenia assessed by QCT technology and the ratio of liver/spleen CT values obtained by conventional CT, in order to clarify the clinical application value of quantitative CT in the diagnosis of fatty liver in patients with schizophrenia.

The rest of this paper is organized as follows: Section 2 discusses related work, followed by the introduction of materials and methods in Section 3.  Section 4 shows the inspection results, and Section 5 concludes the full text primary coverage, major point, and future research directions.

## 2. Related Work

Fatty liver is the most common liver disease characterized by steatosis and lipid deposition of liver parenchymal cells. China fatty liver treatment guidelines (SCIENCE EDITION) show that [4] the prevalence of fatty liver in adults in China reaches 12.5% to 35.4%, exceeding hepatitis B. Fatty liver is easily associated with diabetes and cardiovascular and cerebrovascular diseases [5] and easily induces liver injury, liver fibrosis, cirrhosis, and so on. Because the liver is an organ without pain nerves, its health is often overlooked. The study shows that schizophrenic patients have an unhealthy lifestyle [6], low content of cellulose in their diet and high content of fat, and less exercise at ordinary times. In addition, antipsychotics may have an impact on the liver. Their prevalence of fatty liver is higher than that of ordinary people, which often induces the occurrence of metabolic syndrome and increases the risk of death. Therefore, the accurate diagnosis and classification of fatty liver is conducive to early intervention and can improve the quality of life and survival rate of schizophrenic patients.

RETRACTED

Liver biopsy is the gold standard of hepatic steatosis, but it is not suitable for the screening and repeated follow-up monitoring and evaluation of fatty liver, because it is an invasive examination of focal puncture, which can produce complications such as bleeding and infection [7]. Although ultrasound examination is noninvasive, safe, and radiation-free, the examination results depend more on the performance of ultrasound equipment and doctors' technology and experience. So, its subjective judgment factors are large, and it is relatively insensitive to individuals with liver fat content less than 20% [8]. MRI can make direct quantitative analysis of intrahepatic fat. The examination results are accurate, noninvasive, safe, efficient, and radiation-free. It is of positive significance for the evaluation of patients with fatty liver before and after treatment. However, because our research object is schizophrenic patients, the tolerance and cooperation of them are poor compared with ordinary people, and the MRI examination space is closed, the examination time is long, and the noise is large, so that the results are in a low success rate. The image quality obtained is affected, which will seriously interfere with the accuracy of diagnosis. CT has been proved to be a noninvasive and practical method, which can be used for the quantitative diagnosis of hepatic steatosis, the evaluation of the existence of hepatic fat, and the classification of the severity of fatty liver. Steatosis leads to the attenuation of the liver CT value, which is characterized by the decrease of liver parenchyma density. At the same time, the ratio of the CT value to the spleen CT value can be used for the evaluation of steatosis can also be a clinically practical index for predicting liver fat content and has high specificity for the diagnosis of moderate and severe liver steatosis [9]. Since there is no fat in the spleen, this method has high reliability [10]. At the same time, due to the particularity of schizophrenic patients, it is difficult to ask the medical history and poor tolerance; CT has become the primary imaging method for the examination of abdominal diseases. It is meaningful to evaluate the degree of steatosis without adding additional radiation during abdominal examination. However, the ratio of liver/spleen CT value is a semiquantitative method, which cannot accurately measure the liver fat content. QCT is a new imaging technique for quantitative evaluation of fat content in the liver. The working principle of QCT is to treat the liver as a mixture of pure fat and pure liver tissue, which can be converted into H_2_O and K_2_HPO4 through a certain proportion, and the CT value of ROI can be measured, while the CT value of ROI can be converted into the volume ratio of pure fat and pure liver tissue through phantom conversion and formula [11].

RETRACTED

## 3. Materials and Methods

### 3.1. General Information

The subjects of this study are 457 patients with schizophrenia, who underwent abdominal CT examination in our hospital and QCT examination procedure from June 2020 to December 2021 (according to the fifth edition of the American Diagnostic and Statistical Manual of Mental Disorders (DSM. -V) Diagnostic Criteria for Schizophrenia). Their age ranges from 13 to 90 years old, with an average of 60.67 ± 15.29 years, and 273 males and 184 females. Exclusion criteria are pregnant women, patients with thoracolumbar spine metal implantation, liver lobectomy, splenectomy, liver space-occupying lesions (except benign small cysts and small intrahepatic calcifications), liver cirrhosis, history of alcoholism, and history of hemochromatosis. In addition, the patient is not taking any lipid-lowering drugs or drugs that might cause steatosis (except for second-generation antipsychotics). All subjects obtain informed consent before examination.

### 3.2. Inspection Method

#### 3.2.1. QCT Prescan

A China United Imaging 64-Row uCT 760 Helical CT Scanner is used, and a QCT volume template from MINDWAYS (Mindways Software Inc, Austin, TX, USA) is placed at the center of the scanning bed. Before scanning, the QA phantom and the scanner positioning line are used to guide the adjustment. The position of the QCT volume template and the height of the scan bed is determined, and its position is then fixed as a scan reference. The QA phantom is placed vertically on the QCT phantom, and the conventional CT plain scan is used according to the precalculated height of the scanning bed. The scanning conditions are tube voltage 120 kV, tube current 200 mA, arena rotation speed 0.5s/circle, and pitch 1.0875. The collimation width is 40 cm, the field of view is 500 mm, the layer thickness is 3 mm, and the layer spacing is 3 mm. The reconstruction parameters are standard algorithms, the slice thickness is 1.5 mm, the slice spacing is 1 mm, and the field of view is 500 mm. Upload the reconstructed image to PACS and import it into the MINDWAYS bone density measurement software (QCT Pro version 6.1) workstation, use the software QA Exam function to calibrate the accuracy of the software, and obtain calibration coefficients [12].

#### 3.2.2. CT Examination

Using China United Imaging 64-Slice uCT 760 Helical CT Scanner, the scanning bed is adjusted to the bed height obtained from the prescan, so that the upper abdomen of the patients is located in the center of the QCT volume template and the upper abdomen CT scanning is performed. All patients are in supine position, head first, bilateral upper limbs are raised under calm breathing, and breath is hold to complete the scanning. The scanning parameters are the same as those of the QCT prescan.

RETRACTED

#### 3.2.3. Data Measurement and Analysis

Liver fat content is measured using MINDWAYS bone densitometry software (QCT Pro version 6.1). The software directly measures liver fat content in regions of interest (ROI) in the liver parenchyma based on Hounsfield units and data from a calibrated model. Four ROIs are selected on the liver image of each patient, three ROIs for the right liver and one ROI for the left liver. According to the Glisson system, the liver is divided into 8 segments. ROI 1 is selected for the S8 segment of the right hepatic lobe, and ROI 2, S5, and S6 are selected for the S7 segment. ROI 3 is selected within the region. The left hepatic lobe is usually small in volume, and the layer with the largest left lobe cross-sectional area is selected as ROI 4 in the left hepatic lobe region. The area of each ROI is 300 mm^2^ (±10 mm^2^) as shown in Figure 1. When selecting the ROI, the interference of intrahepatic blood vessels, bile ducts, intrahepatic calcifications, hepatic cysts, ribs, and air in the lungs or gastrointestinal tracta must be avoided. In case of nonuniform fatty liver, it is also measured according to the above standards. For fatty liver patients whose hepatic blood vessels are obliterated and cannot be distinguished, the area close to the liver surface is selected to select ROI. The four measured ROIs are averaged as the final QCT measurement result [12].

The size and position of the four ROIs of the liver and spleen ratio are matched as accurately as possible with the quantitative CT images. At the same time, two equal distance slices of the spleen and spleen hilum are selected to measure the CT values. The measurement results are represented by Hu, and the CT value ratio of the liver/spleen is recorded.

### 3.3. Statistical Analysis

The experimental results are expressed as mean ± standard deviation. Statistical analysis is performed using SPSS 25.0 software. The ratio of the mean liver fat content and the liver/spleen CT value is analyzed by Pearson correlation. The correlation coefficient between groups is evaluated and its consistency is calculated. The ROC subject working characteristic curve is used to analyze the cutoff value of target indexes and evaluate the diagnostic efficiency; inspection level (*α*) is 0.05.

RETRACTED

## 4. Inspection Results

The clinical and imaging parameters of the study population (patients with schizophrenia) are shown in Table 1. The study includes 457 subjects, 273 males (59.74%) and 184 females (40.26%).  Figure 2 is the Pearson correlation between mean liver fat content and liver/spleen CT value ratio. The results of measurement analysis show that the mean liver fat content in all patients had a high negative correlation with the ratio of liver/spleen CT values (*r* = −0.935, *P* < 0.05). Using the ratio of the liver to the spleen as the standard, the ROC curve of liver fat content is drawn to evaluate normal liver and mild fatty liver.

The sensitivity, specificity, and ROC curve of the mean value of liver fat content are shown in Table 2 and Figure 3. The cutoff value of the mean liver fat content between normal liver and mild fatty liver is 9.35%. The sensitivity, specificity, Youden index, and ROC curve of the mean value of liver fat content in mild and moderate fatty liver are shown in Table 3 and Figure 4. The mean cutoff value of fat content in mild and moderate fatty liver is 19.4%, and the sensitivity and specificity are 1 and 1. Because the number of cases of mild and moderate fatty liver is small, this perfect cutoff value appears, and the sensitivity and specificity are 100%.

457 patients are evaluated for fatty liver and grading according to the following three criteria.

1. The liver/spleen ratio standard formulated by the Chinese Society of Hepatology includes two items [13]. The ratio of CT values of the liver and spleen is > 0.7, and <1.0 was considered mild. Degree of fatty liver > 0.5 and ≤ 0.7 is moderate fatty liver and ≤ 0.5 is severe fatty liver.
2. The evaluation standard of American QCT (value conversion refers to the PDFF standard of MRI) is as follows: the mean liver fat content (<5%) is normal, the mean liver fat content (≥5% and <14%) is mild fatty liver, and liver fat content (≥14% and <28%) is moderate fatty liver, and the mean liver fat content (≥28%) is severe fatty liver [14].
3. The data of this study obtains the cutoff value of the mean liver fat content of QCT in patients with schizophrenia, thereby redefining the standard of fatty liver in patients with schizophrenia as follows: the mean liver fat content (<9.35%) is normal, and the mean liver fat content (≥9.35%, <19.4%) is mild fatty liver, mean liver fat content (≥19.4%, <28%) is moderate fatty liver, and mean liver fat content (≥28%) is severe fatty liver.

It is worth noting that this study adopts the liver/spleen CT value ratio standard published by the Chinese Medical Association and the American fatty liver and grading evaluation standard of QCT. When detecting mild fatty liver, the number percentage of mild fatty liver obtained by QCT standard (233/457, 50.98%) is 4 times higher than that obtained by the liver/spleen CT value ratio (57/457, 12.47%). Such a large difference means that the American standard is not accurate or applicable to the Chinese population. Based on the data of schizophrenic patients in this study and the ROC curve drawn with the liver/spleen ratio formulated by the branch of Hepatology of Chinese Medical Association as the reference standard, the new mean value of QCT liver fat content is 9.35% and 19.4% among the diagnosis of normal liver (<9.35%), mild fatty liver (≥9.35%, <19.4%), and moderate fatty liver (≥19.4%, <28%). There is a difference of about 5% compared with the cutoff value of 5% and 14% obtained by QCT American Standard (see Table 4). The reason for the difference between the two standards may be due to the difference in body size between Chinese and American races [15]. Westerners may be larger than Asians as a whole, and the standard identification of fatty liver may be stricter than that in China. Therefore, it is very important to formulate China's own diagnostic criteria of QCT (liver fat content threshold). The percentages of the three evaluation criteria are shown in Table 4.

RETRACTED

## 5. Conclusion

In this study, the average percentage of liver fat content measured by QCT is used to evaluate the degeneration and severity of fatty liver through three different diagnostic and grading criteria of fatty liver, and the differences under different diagnostic criteria are compared. The results of this study show that there is a high correlation between the average percentage of liver fat content and the ratio of liver/spleen CT value in all schizophrenic patients, indicating that QCT is highly feasible in the quantitative diagnosis of fatty liver.

Through the data analysis of this study, it is preliminarily considered that the classification standard of QCT in China is about 5 percentage points higher than that in the United States. It is believed that with further research, the expansion of sample size and the comparison of various populations, a more accurate QCT fatty liver classification diagnostic standard belonging to the Chinese population can be formulated in the future. This study has some limitations. First, because the liver biopsy is invasive and the compliance of schizophrenic patients is poor, all patients do not undergo pathological examination. Second, there are few patients with moderate and severe fatty liver, especially patients with severe fatty liver. The data of such patients need to be further accumulated and analyzed.

RETRACTED

## Figures and Tables

**Figure 1:** The four measured ROIs by QCT: (a) ROI 1, (b) ROI 2, (c) ROI 3, and (d) ROI 4.

**Figure 2:** Pearson correlation between mean liver fat content and liver/spleen CT value ratio.

**Figure 3:** ROC curve of normal liver and mild fatty liver.

**Figure 4:** ROC curve of mild and moderate fatty liver.

**Table 1:** Clinical and imaging parameters of patients with schizophrenia.

Feature	Schizophrenic patients (*n* = 457)
Sex ratio (male:female)	273 : 184 (≈1.5)
Age	60.67 ± 15.29 (13～90)
Height (cm)	165.07 ± 8 .61 (142～182)
Weight (kg)	65.22 ± 12.26 (40～100)
Mean liver fat content (%)	6.83 ± 5.67 (−3.5～50.5)
Liver and spleen CT ratio	1.15 ± 0.20 (−0.38～1.56)

**Table 2:** The relevant index parameters of the ROC curve of normal and mild fatty liver.

Index	AUC	SE	*P*	95% CI	Cutoff value (%)	Sensitivity	Specificity	Youden index
Mean value（%）	0.991	0.004	＜0.001	0.982–1.000	9.35	0.962	0.943	0.905

**Table 3:** The relevant index parameters of the ROC curve of mild and moderate fatty liver.

Index	AUC	SE	*P*	95% CI	Cutoff value (%)	Sensitivity	Specificity	Youden index
Mean value (%)	1.000	0.000	＜0.001	1.000–1.000	19.4	1.000	1.000	1.000

**Table 4:** Percentage of people under different fatty liver assessment criteria.

Criteria and indicators of fatty liver grading		Number of people (*n* = 457)	Percentage (%)
Chinese standard	Liver -spleen ratio (≥1), normal liver	381	83.37
	Liver-spleen ratio (>0.7, <1), mild fatty liver	57	12.47
	Liver-spleen ratio (>0.5, ≤0.7), moderate fatty liver	15	3.28
	Liver-spleen ratio (≤0.5), severe fatty liver	4	0.88

U.S.A QCT standard	Mean liver fat content (<5%), normal liver	184	40.26
	Mean liver fat content (≥5% and <14%), mild fatty liver	233	50.98
	Mean liver fat content (≥14% and <28%), moderate fatty liver	37	8.1
	Mean liver fat content (≥28%), severe fatty liver	3	0.66

Criteria for this study	Mean liver fat content (<9.35%), normal liver	365	79.87
	Mean liver fat content (≥9.35% and <19.4%), mild fatty liver	73	15.97
	Mean liver fat content (≥19.4% and <28%), moderate fatty liver	16	3.5
	Mean liver fat content (≥28%), severe fatty liver	3	0.66

## Data Availability

The simulation experiment data used to support the findings of this study are available from the corresponding author upon request.
